The article "Effect Analysis of Positive Molecular Therapy in Surgical Nursing Based on Data Transformation Analysis" was published in 2022. Journal: Comput Math Methods Med.

# Effect Analysis of Positive Molecular Therapy in Surgical Nursing Based on Data Transformation Analysis

**DOI:** 10.1155/2022/3548854

**Published:** 2022-07-01

**Authors:** Yuan Liu, Sumei Wu, Guifen Wang, Xiaoxue Sun, Lei Liu, Yaling Zhao

**Affiliations:** Department of Cardiothoracic Surgery, Tangshan People's Hospital of Hebei Province, Tangshan, Hebei 063000, China

## Abstract

This paper briefly introduces the concept, classification, and mechanism of action of positive thinking therapy; reviews the application and research progress of positive thinking therapy in perioperative care of surgical patients at home and abroad; presents the shortcomings and defects in the development; and aims to provide intervention, reference, and basis for the development of positive thinking therapy in perioperative care of surgical patients. One hundred and eight patients are undergoing PCI surgery in our cardiology department; 50 patients undergoing percutaneous coronary intervention were selected as the control group, and 58 patients undergoing percutaneous coronary intervention were selected as the observation group. Traditional health education was employed in the control group, while empowerment education based on timing theory was used in the observation group. The two groups were observed and compared in terms of self-care competence, anxiety and depression, medication adherence score, and exercise adherence. *Conclusion*. Empowerment education based on timing theory can improve self-care ability of PCI patients, reduce patients' anxiety and depression, and improve patients' medication and exercise compliance.

## 1. Introduction

With the development of modern medical technology, surgical treatment has become a common method of treatment for various surgical diseases, and quality perioperative management provides an important guarantee for the success of surgery and the patient's future recovery. Most patients face surgery with anxiety, fear, and other adverse emotions due to concerns about the surgical outcome and recovery, causing adverse reactions of the body such as increased heart rate, elevated blood pressure, and flushing, thus affecting the surgical treatment and postoperative recovery [1]. As the scope of medical exploration continues to expand, “positive thinking intervention,” which is an extension of psychology, has been gradually used in clinical research. In recent years, interventions based on positive thinking, such as meditation and stress reduction, have been used in the perioperative period to guide patients to face negative emotional disturbances objectively, relieve psychological stress, and reduce postoperative pain, which play an important role in the operation and postoperative recovery [2]. In this paper, we review the relevant studies at home and abroad and aim to provide reference for the future application of positive thinking therapy in the perioperative period.

The article "Effect Analysis of Positive Molecular Therapy in Surgical Nursing Based on Data Transformation Analysis" was published in 2022. Journal: Comput Math Methods Med.

Since the introduction of positive thinking, psychologists and medical doctors have removed its religious components and applied it to clinical practice. Among them, MBSR and MBCT are the most commonly used, and MBSR and MBCT are currently the most mature and systematic positive thinking interventions [3]. Overseas traditional MBSR and MBCT are group training courses, mostly using the intervention method created by Kabat-Zinn that has a strict training cycle and training courses, the training cycle is generally 8 weeks, once a week, 2.5~3 h each time, and each week there are different types of training methods and coursework, and requires the course instructor to have professional knowledge and skills [4]. In recent years, China has introduced positive thinking into the medical field, in cardiovascular disease, diabetes, cancer, and other clinical diseases to explore, but its adopted treatment is slightly different from foreign countries; the whole course of treatment is 8 weeks, once a week, each time 2.5-3.5 h, requiring 45 min of formal practice and about 10 min of informal practice every day, and in the 6th week a full day retreat (7.5 h). With the continuous improvement of the concept of positive thinking, DBT and ACT have been gradually promoted in clinical practice in recent years and are now mainly used in the treatment of patients with psychiatric disorders such as borderline personality disorder. DBT and ACT can help them to improve their tolerance of negative feelings, reduce behavioral impulses, and enhance their ability to cope effectively with illness [5]. As an important method of psychological treatment for psychological disorders, positive thinking therapy has also played a key role in promoting patients' physical and mental health in clinical practice [6]. Domestic and international studies have shown that the interventions of positive thinking therapy in hypertension, diabetes, chronic pain, cancer, chronic inflammation, and perioperative patients can effectively relieve patients' physical pain, improve patients' emotional disorders, reduce psychological stress, and improve the quality of daily life, which have shown good results in clinical application [7].

Surgery is an invasive treatment, and as a serious source of psychological stress, it can adversely affect the patient's nervous system, endocrine system, and circulatory system, etc. The preoperative stress and anxiety and postoperative physiological trauma can also directly affect the patient's normal physiological activities [8, 9]. In order to solve the psychophysiological problems of patients, clinical workers need to adopt various ways to alleviate the various adverse reactions of patients in the perioperative period [10]. Currently, positive thinking therapies are implemented in the perioperative period in the form of body scans, positive breathing, positive meditation, walking meditation, and positive yoga. Most patients experience anxiety and depression as a result of the invasive nature of surgery and their own stress reactions. Some studies have found that anxiety and depression can increase sympathetic nerve tone and catecholamine secretion, which can cause palpitations, chest tightness, and even a sense of dying, which can seriously affect the operation and postoperative recovery [11]. In recent years, positive thinking therapy has been gradually applied to the guidance of perioperative management of surgical patients. In [12], an 8-week course of standard positive mindfulness stress reduction (tmbsr) was applied to patients awaiting renal transplantation via teleconferencing, and the results showed that TMBSR was effective in helping patients to reduce their preoperative anxiety and discomfort. In a controlled trial of perioperative orthostatic stress reduction therapy in 200 patients undergoing elective surgery, [13] showed that the preoperative systolic blood pressure and heart rate were more stable in the observation group (102 patients) than in the control group (98 patients), and the preoperative anxiety and depression scores in the observation group were significantly lower than those in the control group, which is consistent with the study by [14] and others.

The article "Effect Analysis of Positive Molecular Therapy in Surgical Nursing Based on Data Transformation Analysis" was published in 2022. Journal: Comput Math Methods Med.

The team of [15] used positive meditation training combined with guided psychology on perioperative patients in general surgery and found that the positive meditation training improved the positive thinking ability and positive thinking state of perioperative patients in general surgery, allowing them to better control their negative emotions and psychological reactions. Positive meditation therapy can improve negative psychology and regulate body state for preoperative patients, according to the findings of the above study [16]. At present, China is facing the problems of large medical population, shortage of medical resources, shortage of medical and nursing staff, lack of comprehensive attention to patients' psychological problems, etc. Positive thinking therapy is simple, green, and can compensate for the shortage of medical and nursing staff to a certain extent and can improve the psychological intervention of medical and nursing staff to patients, which has good clinical feasibility [17]. However, the sample size of current studies is generally small, and there is a lack of high quality and standard randomized controlled trials, and the effectiveness of orthomolecular therapy for different surgical diseases remains to be investigated.

The article "Effect Analysis of Positive Molecular Therapy in Surgical Nursing Based on Data Transformation Analysis" was published in 2022. Journal: Comput Math Methods Med.

The research is organized as follows: the optimization algorithms are presented in Section 2.  Section 3 analyzes some of the linear optimization problem.  Section 4 discusses the study subjects. In Section 5, results and discussion were explored in depth.  Section 6 proposed the discussion. Finally, in Section 7, the research work is concluded.

## 2. Optimization Algorithms

### 2.1. Standard Particle Swarm Algorithm

Let the current position and velocity of the *i*th particle of population size *N* be *X*_*i*_ = (*x*_*i*1_, *x*_*i*2_, ⋯, *x*_*iD*_) and *a*_*j*_ ≤ *b*_*j*_, *V*_*i*_ = (*v*_*i*1_, *v*_*i*2_, ⋯, *v*_*iD*_), respectively, and the best position of its current search is *p*_best_, and the best position of all subcurrent searches is *g*_best_. The *j*th dimensional state (1 ≤ *j* ≤ *n*) of the *k* + 1th iteration of particles is updated according to the following formula:

(1) $$\begin{array}{c} v_{ij}^{k+1}=\omega v_{ij}^{k}+C_{1}R_{1}\left(p_{\text{best}}-x_{ij}^{k}\right)+C_{2}R_{2}\left(g_{{\text{bess}}_{ij}}-x_{ij}^{k}\right), \end{array}$$

(2) $$\begin{array}{c} x_{ij}^{k+1}=x_{ij}^{k}+v_{ij}^{k}, \end{array}$$

(3) $$\begin{array}{c} \left\{\begin{array}{c} v_{ij}^{k+1}=v_{\max},\text{if }v_{ij}^{k+1}>v_{\max},\\ v_{ij}^{k+1}=-v_{\max},\text{if }v_{ij}^{k+1}<-v_{\max}, \end{array}\right. \end{array}$$

(4) $$\begin{array}{c} \left\{\begin{array}{c} {x_{ij}}^{k+1}=a_{j},{{ifx}_{ij}}^{k+1}<a_{j},\\ {x_{ij}}^{k+1}=b_{j},{{ifx}_{ij}}^{k+1}>b_{j}, \end{array}\right. \end{array}$$

where *i* = 1, 2, ⋯*N*, *j* = 1, 2, ⋯*D*.

Parameter description *ω* is called the inertia weight, which determines the influence of the particle historical velocity information current velocity information. *C*_1_, *C*_2_ is called the learning factor, which indicates the degree to which the particle is influenced by individual cognition and social cognition, and is usually set to *C*_1_ = *C*_2_ = 2. *R*_1_, *R*_2_ indicates a random number uniformly distributed between [0.1]. In addition, the particle *i* is constantly adjusting its position according to the velocity and is limited by the maximum velocity *v*_max_ which is usually set to 10%-100% of the variation range per dimension.

### 2.2. Monte Carlo Algorithm

The Monte Carlo approach, also known as random simulation (Randulation), is a series of numerical methods for solving nonlinear problems. It is derived from the random process of roulette and coin tossing. The principle of Monte Carlo algorithm is as follows: statistical experiments and random simulation as a means, from the probability distribution of random variables through the method of randomly selected numbers, to produce a random sequence of numbers consistent with the characteristics of the probability distribution of the random variables, as the infant sequence for simulation.

The article "Effect Analysis of Positive Molecular Therapy in Surgical Nursing Based on Data Transformation Analysis" was published in 2022. Journal: Comput Math Methods Med.

## 3. Linear Optimization Problem

The first and second steps of the calibration of the nonlinear visual model are performed separately for the linear initial value solution and the initial nonlinear optimization of the NIE model, respectively. The parameters of the calibration are optimized in the process. According to the camera model, from the known object feature points projected onto the image plane, the model image coordinates of the feature points(*U*_*i*_, *V*_*i*_), the model image coordinates(*U*_*i*_, *V*_*i*_)and the actual camera detected image coordinates, and there are residuals; the purpose of nonlinear optimization is to minimize this residual, so that the parameters minimize the residuals for the camera parameter values. The analytical expression of the objective function of the optimization is

(5) $$\begin{array}{c} F=\min\overset{n}{\underset{i=1}{\sum }}\overset{n}{\underset{j=1}{\sum }}d{\left(Q\left(a_{j},b_{j}\right),x_{ij}\right)}^{2}, \end{array}$$

where *x*_*ij*_ denotes the 2D image point coordinates of the *i*th spatial point on the first picture, which is extracted directly from the image. *Q*(*a*_*j*_, *b*_*j*_) is the projected coordinates obtained by taking the known 3D point scale and the external parameter values, according to the projection relation. *a*_*j*_ denotes the first picture, and *b*_*j*_ denotes the coordinates of the *i*th 3D point. *d*(*x*, *y*) denotes the Euclidean distance of these two *x*, *y* vectors. The goal of the optimization is to minimize the residuals of the 2D coordinates obtained by these two different paths.

### 3.1. Algorithm Flow

The MPSO algorithm steps are as follows: the algorithm uses linear decreasing weight particle swarm for rough search at the early stage of evolution and improves the solution accuracy by using Monte Carlo algorithm for random search at the later stage.

**Step 1 .**

The particle population (population size in *N*) for each particle in the initialization range for the speed and position of random initialization to ensure population variety, all particle positions uniformly distributed in the search area particle positions are initialized according to the following formula:

(6) $$\begin{array}{c} x_{ij}=a_{j}+\left(i-1\right)\times \left(b_{j}-a_{j}\right)/N+\left(\left(b_{j}-a_{j}\right)/N\right)\times R, \end{array}$$

where *R* is the random number *i* = 1, 2, ⋯, *N*, *j* = 1, 2, ⋯*D* evenly distributed between [0,1].

The article "Effect Analysis of Positive Molecular Therapy in Surgical Nursing Based on Data Transformation Analysis" was published in 2022. Journal: Comput Math Methods Med.

**Step 2 .**

Calculate the adaptation values of all particles.

**Step 3 .**

Update the best position *p*_best_ experienced by each particle and the best position *g*_best_ experienced by all particles according to the current state of the particle population.

**Step 4 .**

Calculate the inertia weights according to equation (7) to update the velocity and position of particles according to equations (8) and (2), and use equations (3) and (4) to cross the boundary.

(7) $$\begin{array}{c} \omega^{k}=\omega_{\max}-\left(\left(\omega_{\max}-\omega_{\min}\right)/{it}_{\max}\right)\times k, \end{array}$$

(8) $$\begin{array}{c} {v_{ij}}^{k+1}=\omega^{k}{v_{ij}}^{k}+C_{1}R_{1}\left(p_{\text{bert}ij}-{x_{ij}}^{k}\right)+C_{2}R_{2}\left(g_{\text{best }ij}-{x_{ij}}^{k}\right). \end{array}$$

**Step 5 .**

When the number of iterations does not reach the maximum number of iterations *it*_max_, then go to Step 2; if it reaches the maximum number of iterations, then go to Step 6.

**Step 6 .**

Make *j* = 1 and *j* < 10^4^, *k* = 1, *m*_1_ = *m*_2_ = ⋯*m*_*D*_ = 1, *x*^*j*^ = *g*_*best*_ = (*x*_1_^*j*^, *x*_2_^*j*^, ⋯, *x*_*d*_^*j*^), *B*_*i*_ = (*b*(*i*) − *a*(*i*)), *i* = 1, 2, ⋯, *D*, *F*_1_ = *f*(*x*^*j*^).

**Step 7 .**

*m*_*k*_ = *m*_*k*_ + 1, if *m*_*k*_ > 10^5^,and *B*_*k*_ > *ε*, so that *B*_*k*_ = *B*_*k*_/2, *m*_*k*_ = 0.

**Step 8 .**

Generate a random number *x*_*k*_^*j*^ = *x*_*k*_^*j*−1^ + *r*_*k*_^*j*^, *F*_2_ ≥ *F*_1_ = *F*(*x*^*j*^) according to uniform distribution on (−*B*_*k*_, *B*_*k*_), make *x*_*k*_^*j*^ = *x*_*k*_^*j*−1^ + *r*_*k*_^*j*^, and calculate *F*_2_ = *F*(*x*^*j*^); if*F*_2_ ≥ *F*_1_, make *x*_*k*_^*j*^ = *x*_*k*_^*j*^ − *r*_*k*_^*j*^, , and return to Step 7; otherwise, make *F*_2_ = *F*_,_*k* = *k* + 1; if *K* > *D*, make *k* = 1, *j* = *j* + 1, *x*_*k*_^*j*^ = *x*_*k*_^*j*−1^, *k* = 1, 2, ⋯, *D*.

**Step 9 .**

Check whether the preset precision *ε* and the maximum number of iterations are reached, if not, and *j* < 10^4^, then return to Step 7; otherwise, *x*^*j*^ = (*x*_1_^*j*^, *x*_2_^*j*^, ⋯, *x*_*D*_^*j*^) will be the final value of *F* solution.

## 4. Study Subjects

Patients undergoing percutaneous coronary intervention in the cardiology department of our hospital were selected as the study subjects. Inclusion criteria are as follows: (1) confirmed diagnosis of coronary artery disease, (2) good understanding and communication skills, and (3) informed consent of the patients and their families and willingness to cooperate with this study. Exclusion criteria are as follows: (1) combined with other cardiac diseases other than coronary heart disease; (2) suffering from cognitive dysfunction or psychological or psychiatric diseases; (3) combined with other serious physical diseases such as tumor, liver, and kidney insufficiency; and (4) patients with joint, muscle, neurological, and other diseases that cannot cooperate with exercise rehabilitation. Exclusion criteria are as follows: (1) only contrast surgery that was performed on patients who did not fit the criteria for PCI procedure; (2) postoperative complications such as bleeding, restenosis, and occlusion of the implanted stent after PCI; and (3) patients who withdrew voluntarily. The final 108 patients were included in the study, 50 patients with percutaneous coronary intervention in March-May 2019 as the control group and 58 patients with percutaneous coronary intervention in June-August 2019 as the observation group. There was no statistically significant difference between the general data of the 2 groups such as gender, age, education, smoking history, drinking history, and number of stents (*P* > 0.05). The details are shown in Table 1.

The article "Effect Analysis of Positive Molecular Therapy in Surgical Nursing Based on Data Transformation Analysis" was published in 2022. Journal: Comput Math Methods Med.

### 4.1. Methods

A total of four face-to-face health education sessions were conducted during hospitalization, each for about 30 min. They were carried out by charge nurses with clinical experience and were identical to those in the observation group. Patients and family members received information regarding coronary heart disease and general health education materials on the day of admission; 1 day before surgery, the process and preoperative preparation were explained, and patients were taught psychological relaxation techniques; on the day after surgery, skin care at the puncture site, the importance of postoperative medication; the effects of aspirin, clopidogrel, and other drugs; and the observation and treatment of adverse reactions were introduced; 1 d before discharge, a manual on rehabilitation exercises was distributed. Patients were followed up by telephone once a month for 3 months. The follow-up included the implementation of rehabilitation exercises, diet, medication standardization, and self-monitoring of diseases such as blood pressure and blood glucose.

### 4.2. Observation Group

Empowerment education research group was established including the director of the cardiology department (professor and master's supervisor), the head nurse (supervising nurse with more than 20 years of clinical work experience), 3 charge nurses (with more than 10 years of cardiology nursing experience), 2 nurses of the cardiac rehabilitation center (with provincial specialist nurse certificate), 2 nursing master students, and 1 psychological counselor (with national level 2 psychological counselor certificate). All team members underwent standardized training and passed the examination and were proficient in the intervention process.

The article "Effect Analysis of Positive Molecular Therapy in Surgical Nursing Based on Data Transformation Analysis" was published in 2022. Journal: Comput Math Methods Med.

The timing theory illness stage division was used as a reference in this investigation. To establish the intervention strategy for this study, the team members conducted a local and international literature search, clinical investigation with the features of PCI patients, expert consultation, and preexperimentation. This includes (1) the division of disease stages: diagnostic period (from disease onset to definite diagnosis), PCI perioperative period (patient's decision to operate to postoperative stabilization), discharge preparation period (patient's treatment is about to end to discharge), adjustment period (after discharge to 1 month), and adaptation period (1 month to 3 months after discharge). (2) Determining the content of empowerment education includes as follows: (a) For question identification, the interventionist uses in-depth conversation with the patient using empathy and emotional support, asks the patient targeted questions, and understands the patient's current needs based on the patient's responses. (b) For emotional expression, start with an open-ended topic, induce the patient to tell or vent his emotions, do not interrupt the patient easily, pay attention to listening and responding at the right time, and explore the patient's innermost emotions. (c) For goal setting, group members act as a supporting role, actively provide medical information to support the patient, and the patient proposes goals. Team members help analyze the feasibility of the goals according to the patient's actual situation and make adjustments if necessary. (d) Develop a plan, in which the researcher helps the patient to develop a health promotion plan based on the set goals, and the patient chooses the method that meets his or her wishes. The main purpose of the program is to teach the researcher the relevant knowledge, the patient's participation in the discussion, and the training of relevant coping skills. (e) Behavioral assessments were carried out on a regular basis to track the improvement of patients and their families. If the goals are not met, actively seek out the reasons and make changes as soon as possible to boost the patient's self-esteem and treatment compliance.

The intervention was carried out by the investigator herself and a uniformly trained specialist nurse from the study team, with team members supervising throughout. The intervention was divided into in-hospital interventions: the diagnostic period, the PCI perioperative period, and the discharge preparation period. The intervention time was mainly focused around 20 : 00. The interventions were conducted 1 to 2 times per phase, each time for 30 to 45 min. The interventions were conducted in a face-to-face one-to-one format, mainly in the departmental demonstration room. Out-of-hospital interventions include adjustment and adaptation periods. The intervention time was agreed with the patient in advance, with one telephone follow-up intervention and one home visit per phase. Each visit was 15-30 min.

The article "Effect Analysis of Positive Molecular Therapy in Surgical Nursing Based on Data Transformation Analysis" was published in 2022. Journal: Comput Math Methods Med.

### 4.3. Observation Index

The Exercise of Self-Care Agency (ESCA) scale was developed by the American scholars Kearney and Fleischer in 1979 and is now widely used to test the self-care ability of patients with coronary heart disease in China. Self-concept, self-care responsibility, self-care abilities, and health knowledge are among the 43 items and four dimensions. A 5-point Likert scale was utilized, with a score ranging from “extremely unlike me” to “quite like me.” The higher the total score, the better the patient's ability to care for themselves. The Cronbach *α* coefficient of the English version of the scale was 0.862, which was translated into Chinese by Hsin-Hung in Taiwan. Its Cronbach *α* coefficient was 0.83-0.98. It was assessed before the intervention, at the time of discharge, at the end of 1 month after discharge, and at the end of 3 months after discharge.

The Self-Rating Anxiety Scale (SAS) and the Self-Rating Depression Scale (SDS) developed by Zung et al. were used to assess the subjective feelings of individuals with anxiety/depression tendencies. The 4-point Likert scale was used for both the SAS and the SDS.

#### 4.3.1. Medication Adherence

The Morisky Medication Adherence Questionnaire was developed by Prof. Morisky. This questionnaire was used to measure medication adherence in patients with chronic diseases. There are 8 items, including whether patients forget to take their medication, whether they stop taking their medication or reduce their dose, and whether they carry their medication with them when they go out for a long period of time. A dichotomous scale was used, with a “1/0” score for each “yes/no” answer and a total score of 0 to 8. The higher the score, the better the patient's medication adherence, and the Cronbach *α* coefficient of the scale was 0.72. At discharge, at the end of the first month after discharge, and at the end of the second month after discharge. The assessment was performed at the time of discharge, at the end of 1 month after discharge, and at the end of 3 months after discharge.

The article "Effect Analysis of Positive Molecular Therapy in Surgical Nursing Based on Data Transformation Analysis" was published in 2022. Journal: Comput Math Methods Med.

#### 4.3.2. Exercise Compliance

According to the expert consensus on exercise rehabilitation after PCI, patients were emphasized to exercise at least 3 times per week for at least 30 min each time for 3 months. Patients were considered to be in good compliance if they completed 80 percent or more of the total weekly recommended exercise time, good compliance if they completed 60 percent or more of the total weekly recommended exercise time, and poor compliance if they completed less than 60 percent of the total weekly recommended exercise time. The assessment was recorded at the completion of the intervention.

#### 4.3.3. Data Collection Method

The data were collected by the investigator himself, and the baseline data were collected face-to-face on the day of admission for both groups of patients. The patients' self-care scores, anxiety-depression scores, and medication adherence scores were collected again on the day of discharge, and the patients' self-care scores, anxiety-depression scores, and medication adherence scores were collected by micromail or home visits at 1 month and 3 months of discharge, respectively; and the patients' exercise adherence was evaluated by the exercise diary filled by the patients at 3 months of discharge.

## 5. Results

### 5.1. Comparison of Self-Care Competency Scores

Using repeated measures ANOVA, spherical tests were performed for self-concept, self-care responsibility, self-care skills and health knowledge, and total scores of PCI patients (*W* = 0.232, 0.193, 0.155, 0.205, and 0.039, *P* < 0.001), respectively. Geisser corrected the results, and the patients in the observation group had higher scores on all dimensions and total scores than the control group (*F* = 27.337, 28.998, 14.424, 18.651, and 88.001, *P* < 0.001). The differences in the scores and total scores of the dimensions of self-care competency at different time points were statistically significant (*F* = 242.119, 288.911, 1288.541, 355.205, and 293.233, *P* < 0.001); there was a more reciprocal effect between groups and time (*F* = 109.131, 55.055, 183.819, 101.567, and 70.606, *P* < 0.001). There was no statistically significant difference between the scores and total scores of self-care ability of the two groups before the intervention (*P* > 0.05); there was a statistically significant difference between the scores and total scores of self-care ability of the two groups at discharge, at the end of 1 month after discharge, and at the end of 3 months after discharge (*P* < 0.05). The details are shown in Table 2.

### 5.2. Anxiety and Depression Scores

Anxiety and depression scores of patients are undergoing percutaneous coronary intervention in 2 groups.

The article "Effect Analysis of Positive Molecular Therapy in Surgical Nursing Based on Data Transformation Analysis" was published in 2022. Journal: Comput Math Methods Med.

The Chinese adult anxiety normative score was 28.88 ± 10.19, and the Chinese adult depression normative score was 33.51 ± 8.62, which were lower than the anxiety and depression scores of patients in the 2 groups in this study at each time point, and the differences were statistically significant (*P* < 0.001). See Table 3.

### 5.3. Comparison of Anxiety and Depression

The comparison of anxiety and depression scores between 2 groups of patients is undergoing percutaneous coronary intervention.

First by spherical test (*W* = 0.026 and 0.030, *P* < 0.001), the spherical test was not satisfied (*P* < 0.10). After using the Greenhouse-Geisser correction, the SAS and SDS scores were higher in the observation group than in the control group (*F* = 22.751 and 34.351, *P* < 0.001). The differences in SAS and SDS scores at different time points were statistically significant (*F* = 206.228 and 829.213, *P* < 0.001); there was an interaction between group and time (*F* = 36.111 and 223.733, *P* < 0.001). There was no statistically significant difference between the SAS scores and SDS scores of the 2 groups before the intervention (*P* > 0.05). There was a statistically significant difference between the self-SAS and SDS scores of the two groups at discharge, one month after discharge, and three months after discharge (*P* < 0.05). Details are shown in Table 4.

The sphericity test was first tested (*W* = 0.746, *P* < 0.001), and the sphericity test was not satisfied (*P* < 0.10). The results were corrected using the Greenhouse-Geisser correction, and the patients in the observation group had higher medication adherence than the control group (*F* = 12.235, *P* < 0.001). The difference in scores at different time points was statistically significant (*F* = 58.232, *P* < 0.001); group and time had a more reciprocal effect (*F* = 38.713, *P* < 0.001). There was no statistically significant difference between the scores of the 2 groups at the time of discharge (*P* > 0.05); at the end of 1 month after discharge and at the end of 3 months after discharge, there was a statistically significant difference between the scores of the 2 groups (*P* < 0.05). Details are shown in Table 5.

The comparison of exercise compliance between the 2 groups of patients is undergoing percutaneous coronary intervention. The differences in exercise compliance between the 2 groups of patients were statistically significant (*P* < 0.05), as shown in Table 6.

## 6. Discussion

In postoperative patients, wound pain, tubing restrictions, and concerns about recovery can affect the psychological, physical, and social recovery of patients. The application of positive thinking therapy and progressive muscle relaxation training to postoperative rehabilitation of patients undergoing cardiothoracic surgery was found to be effective in reducing postoperative physical and psychological problems, as well as improving the quality of sleep and psychological mood of patients, according to a study by [18]. In a study by [19], it was concluded that positive stress reduction therapy was effective in reducing perceived stress levels in postoperative breast cancer patients, and [20] confirmed the long-term effects of positive stress therapy in improving postoperative anxiety and depression in breast cancer patients up to 1 year after the intervention. Furthermore, a number of studies have found that incorporating orthomolecular therapy into the postoperative care of patients undergoing surgical procedures such as hip replacement, cranial surgery, and radical esophageal cancer improves patients' perception and orthomolecular level, improves their pain experience, and promotes wound healing, all of which have a positive effect on their recovery. This may be related to the neuromodulation mechanism of orthomolecular therapy, but the details need to be further investigated. The above results suggest that positive thinking therapy has positive significance in promoting postoperative recovery, not only reducing body pain and relieving postoperative psychological stress, but also improving patients' quality of life. However, in most of the studies, the implementers did not receive systematic training in orthomolecular therapy and did not obtain the corresponding qualification, and there is a lack of unified protocols and consistent evaluation indexes in each region and hospital, so it is impossible to accurately understand the patient's compliance and intervention effect [21–24].

The article "Effect Analysis of Positive Molecular Therapy in Surgical Nursing Based on Data Transformation Analysis" was published in 2022. Journal: Comput Math Methods Med.

## 7. Conclusion

Positive thinking therapy, as a new psychological intervention, has played a positive role in promoting perioperative surgery and postoperative recovery. However, due to the small sample size, most of the studies in China are cross-sectional studies with small samples, and there is a lack of postintervention evaluation tools and long-term postoperative follow-up of the patients, which makes it impossible to comprehensively evaluate the intervention effects. Furthermore, the current study's participants were mostly adults, and more research is needed to see if the positive thinking intervention strategy can be used with youngsters. Future studies should increase the sample size and strengthen the follow-up, and we should combine it with the “clown boil method” to conduct trials in children. We should also cultivate a specialized positive thinking intervention team, establish specific local measurement criteria based on the domestic environment, follow up the patients, and evaluate the intervention effect. It should also be fully integrated with the characteristics of hospital departments and patient care in China and be used as a powerful intervention tool to promote the development of positive thinking intervention in clinical practice.

## Figures and Tables

**Table 1:** Comparison of general information of patients in 2 groups with percutaneous coronary intervention.

Group	Observation group (*n* = 58)	Control group (*n* = 50)	Statistic	*P*
Age ($\bar{X\underline{+}S}$ years)	61.33 ± 869	60.92 ± 8.05	*t* = 0.101	0.919
Gender	31	28	*x* ^2^ = 0.015	0.904
Male	27	22		
Female				
Educational level	46	41	*x* ^2^ = 0.749	0.402
High school or below	14	7		
College or above				
Course of disease (years)			*x* ^2^ = 0.588	0.445
≤5	38	38		
>5	18	14		
Disease type			*x* ^2^ = 0.521	0.482
Angina pectoris	27	18		
Myocardial infarction	31	32		
Disease severity			*x* ^2^ = 0.199	0.651
Mild	35	28		
Moderate and severe	24	21		
Number of implanted stents			*x* ^2^ = 0.259	0.611
≤3	33	27		
>3	23	25		
Body mass index			*x* ^2^ = 0.071	0.794
<24	15	10		
≥24	45	38		
Smoking history			*x* ^2^ = 0.028	0.871
Yes	37	33		
No	19	19		
Drinking history			*x* ^2^ = 0.471	0.497
Yes	26	21		
No	32	29		

**Table 2:** Comparison of self-care ability scores of patients with percutaneous coronary intervention in 2 groups ($\bar{X}\pm S$, points).

Group	*n*	Before intervention	At the end of discharge	One month after discharge	Three months after discharge	Total	*F*	*P*
Self-concept								
Observation group	58	14.91 ± 1.60	16.60 ± 1.99	18.23 ± 2.14	19.11 ± 2.08	18.01 ± 1.91	259.382	<0.001
Control group	50	15.63 ± 2.22	15.77 ± 3.14	15.78 ± 3.26	15.29 ± 1.88	15.05 ± 1.04	38.839	<0.001
Total		14.69 ± 2.01	16.07 ± 2.11	17.02 ± 2.63	17.33 ± 2.73	16.51 ± 2.14	242.119	<0.001^#^
*F*		0.933	2.951	6.190	9.651	27.337	109.131	<0.001∗
*P*		0.361	0.004	<0.001	<0.001	0.001^#^		
Sense of self-care responsibility								
Observation group	58	11.52 ± 1.22	13.12 ± 1.02	14.03 ± 1.13	12.09 ± 1.16	10.97 ± 1.36	286.991	<0.001
Control group	50	9.69 ± 1.96	10.13 ± 1.52	10.91 ± 1.41	11.65 ± 1.55	10.69 ± 1.55	48.851	<0.001
Total		9.55 ± 2.12	11.01 ± 1.51	12.09 ± 1.63	12.93 ± 1.86	11.53 ± 1.23	288.911	<0.001^#^
*F*		1.179	5.251	9.335	9.324	28.998	55.055	<0.001∗
*P*		0.240	<0.001	<0.001	<0.001	0.001^#^		
Self-care skills								
Observation group	58	21.61 ± 3.40	23.78 ± 3.01	25.39 ± 4.11	26.51 ± 3.39	24.88 ± 2.57	2829.799	<0.001
Control group	50	21.03 ± 2.38	22.11 ± 2.91	23.19 ± 2.85	23.09 ± 2.85	22.11 ± 2.85	151.737	<0.001
Total		21.41 ± 2.78	22.97 ± 3.11	24.48 ± 3.09	24.93 ± 3.26	23.57 ± 3.02	1288.541	<0.001^#^
*F*		1.132	2.855	4.384	6.381	14.424	183.819	<0.001∗
*P*		0.261	0.049	<0.001	<0.001	0.001^#^		
Health knowledge level								
Observation group	58	25.71 ± 2.21	27.53 ± 2.36	29.37 ± 2.59	30.69 ± 2.81	28.35 ± 2.31	464.733	<0.001
Control group	50	25.37 ± 2.13	25.81 ± 2.13	27.21 ± 2.69	26.45 ± 2.56	26.31 ± 2.51	52.451	<0.001
Total		25.57 ± 3.01	26.39 ± 2.39	28.39 ± 2.89	28.39 ± 3.26	12.36 ± 2.63	355.205	<0.001^#^
*F*		0.743	4.143	4.186	7.222	18.651	101.567	<0.001∗
*P*		0.459	<0.001	<0.001	<0.001	0.001^#^		
Total score								
Observation group	58	71.89 ± 3.86	79.81 ± 6.23	86.53 ± 4.28	89.79 ± 4.25	82.19 ± 4.21	353.555	<0.001
Control group	50	71.23 ± 3.49	74.19 ± 6.11	77.39 ± 5.19	76.87 ± 5.22	77.81 ± 4.96	37.062	<0.001
Total		71.69 ± 3.69	77.14 ± 6.35	82.22 ± 6.59	83.71 ± 7.78	78.39 ± 6.31	293.233	<0.001^#^
*F*		0.888	4.985	10.312	14.711	88.001	170.606	<0.001∗
*P*		0.441	<0.001	<0.001	<0.001	0.001^#^		

Note: # indicates the main effect; ∗ indicates the interaction effect.

The article "Effect Analysis of Positive Molecular Therapy in Surgical Nursing Based on Data Transformation Analysis" was published in 2022. Journal: Comput Math Methods Med.

**Table 3:** Comparison of the anxiety-depression scores of patients with percutaneous coronary intervention in 2 groups with the Chinese adult normative score ($\bar{X}\pm S$, points).

Group	*n*	Before intervention	At the end of discharge	One month after discharge	Three months after discharge
Anxiety score					
Observation group	58	57.44 ± 4.33	55.25 ± 5.29	50.33 ± 5.17	46.61 ± 5.83
Control group	50	57.67 ± 4.32	56.89 ± 3.31	55.69 ± 3.31	53.19 ± 4.38
Norm	1168	28.88 ± 10.19	28.88 ± 10.19	28.88 ± 10.19	28.88 ± 10.19
*t*_1_		30.901	24.798	20.612	16.011
*P*_1_		<0.001	<0.001	<0.001	<0.001
*t*_2_		32.001	32.659	30.712	27.123
*P*_2_		<0.001	<0.001	<0.001	<0.001
Depression score					
Observation group	58	56.39 ± 4.19	54.44 ± 4.32	50.31 ± 4.50	47.98 ± 4.69
Control group	50	56386 ± 4.23	58.03 ± 3.37	56.07 ± 3.34	55.51 ± 3.27
Norm	1355	33.51 ± 8.62	33.51 ± 8.62	33.51 ± 8.62	33.51 ± 8.62
*t*_3_		22.601	19.333	15.991	13.159
*P*_3_		<0.001	<0.001	<0.001	<0.001
*t*_4_		22.687	25.123	23.512	21.457
*P*_4_		<0.001	<0.001	<0.001	<0.001

Note: *t*_1_, *t*_2_ indicates the comparison of SAS observation group and control group with the Chinese adult norm; *t*_3_, *t*_4_ indicates the comparison of SDS observation group and control group with the Chinese adult norm.

**Table 4:** Comparison of anxiety and depression scores between the 2 groups of patients undergoing percutaneous coronary intervention ($\bar{X}\pm S$, points).

Group	*n*	Before intervention	At the end of discharge	One month after discharge	Three months after discharge	Total	*F*	*P*
Anxiety score								
Observation group	58	57.41 ± 4.21	55.12 ± 5.22	50.32 ± 5.33	47.11 ± 5.69	53.09 ± 5.41	209.123	<0.001
Control group	50	57.99 ± 3.98	57.01 ± 3.19	55.63 ± 3.49	54.11 ± 4.31	55.99 ± 5.39	35.889	<0.001
Total		57.59 ± 4.31	55.50 ± 4.61	52.88 ± 5.31	49.68 ± 6.19	54.01 ± 1.13	206.228^#^	<0.001^#^
*F*		0.599	2.858	6.085	6.940	22.751^#^	36.111∗	<0.001∗
*P*		0.539	0.049	<0.001	<0.001	0.001^#^		
Depression score								
Observation group	58	56.29 ± 4.11	54.44 ± 4.29	50.39 ± 4.50	48.11 ± 4.63	52.33 ± 3.39	1104.007	<0.001
Control group	50	57.09 ± 4.26	58.13 ± 3.41	56.08 ± 3.21	54.26 ± 3.30	57.01 ± 3.54	84.001	<0.001
Total		56.66 ± 4.13	55.51 ± 3.39	52.21 ± 5.51	50.82 ± 5.21	54.00 ± 4.13	829.213^#^	<0.001^#^
*F*		0.719	6.342	7.349	8.999	34.351^#^	223.733∗	<0.001∗
*P*		<0.001	<0.001	<0.001	<0.001	0.001^#^		

Note: # indicates the main effect; ∗ indicates the interaction effect.

The article "Effect Analysis of Positive Molecular Therapy in Surgical Nursing Based on Data Transformation Analysis" was published in 2022. Journal: Comput Math Methods Med.

**Table 5:** Comparison of medication adherence scores between the 2 groups of patients undergoing percutaneous coronary intervention ($\bar{X}\pm S$, points).

Group	*n*	At the end of discharge	One month after discharge	Three months after discharge	Total	*F*	*P*
Observation group	58	6.44 ± 0.79	6.69 ± 0.83	6.37 ± 0.88	6.56 ± 0.81	18.537	<0.001
Control group	50	6.51 ± 0.87	6.17 ± 0.99	5.35 ± 0.73	6.04 ± 0.87	51.001	<0.001
Total		6.47 ± 0.86	6.55 ± 0.94	5.91 ± 0.93	6.18 ± 0.99	58.232∗	<0.001^#^
*F*		0.423	3.129	7.311	12.235^#^	38.713∗	<0.001∗
*P*		<0.001	<0.001	<0.001	0.001^#^		

Note: # indicates the main effect; ∗ indicates the interaction effect.

**Table 6:** Comparison of exercise compliance levels between the 2 groups of patients undergoing percutaneous coronary intervention (cases).

Group	*n*	Good	Excellent	Bad
Observation group	58	29	20	9
Control group	50	21	12	17
*Z*			2.089	
*P*	0.037			

## Data Availability

The dataset used in this paper are available from the corresponding author upon request.
